# Synergistic and Attenuating Effect of Electroacupuncture on Aconitine in Improving Heart Failure and Its Calcium Regulation Mechanism

**DOI:** 10.1155/2022/4940745

**Published:** 2022-07-14

**Authors:** Chen Zhou, Mo-Zheng Wu, Qun Liu, Juan-Juan Xin, Shuang Wu, Yu-Xue Zhao, Wen-Xi Zhang, Xiao-Chun Yu, Jun-Hong Gao

**Affiliations:** Institute of Acupuncture and Moxibustion, China Academy of Chinese Medical Sciences, Beijing, China

## Abstract

**Objective:**

The objective is to observe the synergistic and attenuating effect of electroacupuncture (EA) on aconitine (ACO) in improving heart failure (HF) and to explore its underlying mechanism for calcium regulation.

**Methods:**

Twenty-four male Sprague-Dawley rats were randomly divided into four groups: normal control (NC) (*n* = 6), HF(*n* = 6), ACO (*n* = 6), and ACO + EA (*n* = 6). The maximum rates of left ventricular pressure rising and declining (±dp/dtmax), arrhythmia, the left ventricular systolic pressure (LVSP), ejection fraction (LVEF), and fractional shortening (LVFS) were measured by physiological recorder and ultrasound, respectively. Protein expressions of sarcoplasmic/endoplasmic reticulum Ca^2+^ ATPase (SERCA2a), phospholamban (PLB), and Na^+^-Ca^2+^ exchange (NCX1) in the left ventricle tissue were detected by fluorescence immunoblotting.

**Results:**

Compared with the NC group, LVSP, ±dp/dtmax, LVEF, and LVFS were decreased in the HF group; compared with the HF group, LVSP, ±dp/dtmax, LVEF, and LVFS were significantly increased in the ACO + EA group. Compared with the ACO group, the incidence and the degree of arrhythmia were significantly reduced in the ACO + EA group. Compared with the NC group, the activity of SERCA2a was decreased, and the expression of PLB and NCX1 was enhanced in the HF group; compared with the HF group and ACO group, the activity of SERCA2a was increased, and the expression of PLB and NCX1 was significantly attenuated in the ACO + EA group.

**Conclusions:**

EA plays a synergistic and attenuated role in ACO improving HF, and the mechanism may be related to the enhancement of the SERCA2a activity and the decrease of the expression of PLB and NCX1 in cardiomyocytes.

## 1. Introduction

Heart failure is a complex clinical syndrome of impaired ventricular filling or competence due to structural or functional diseases of the heart and is the terminal stage of a variety of cardiovascular diseases [1]. Nowadays, nearly 30 million patients with heart failure worldwide have a five-year survival rate of 50%, which is equivalent to cancer and has become a major disease that seriously affects public health [2, 3]. With the global aging, the prevalence of heart failure is bound to continue to climb. In recent years, although diuretics, *β*-blockers, angiotensin-converting enzyme inhibitors, and other clinical routine medications have achieved clear positive results, they are accompanied by hypotension, renal impairment, electrolyte imbalance, and other side effects. Moreover, long-term use can easily lead to drug resistance [4]. Therefore, how to actively intervene in heart failure is particularly important.

At present, the medical community has focused on the study of heart failure treatment on the calcium cycle defect of sarcoplasmic reticulum (SR) [5]. *Fuzi* as a traditional Chinese medicine has been applied to the treatment of heart failure for thousands of years. However, if the dosage is not appropriate, it can easily cause arrhythmia, so its clinical application is greatly restricted. Recent pharmacological studies have shown that aconitine, a diester diterpene alkaloid, is the main active component of *Fuzi*, and its cardiotonic effect and cardiotoxicity are all related to the mechanism of calcium regulation in cardiomyocytes [6]. On the other hand, a large number of basic studies have confirmed that electroacupuncture can regulate the expression of key proteins of calcium regulation, reduce intracellular calcium ([Ca^2+^]_i_) overload in cardiomyocytes, enhance myocardial contractility, and can improve ischemic arrhythmias with protective effects on the myocardium [7]. In view of this, this study will observe the synergistic and attenuated effect of electroacupuncture on aconitine in improving heart failure, on this basis take the mechanism of calcium regulation in cardiomyocytes as the starting point, and systematically explore its related mechanism of action in order to open up an effective and safe new way for acupuncture combined with medicine in the treatment of heart failure.

## 2. Materials and Methods

### 2.1. Animal Preparation and Animal Grouping

Twenty-four eight-week-old male Sprague-Dawley rats weighing 250–310 g were randomly divided into 4 groups: NC group (*n* = 6), HF group (*n* = 6), ACO group (*n* = 6), and ACO + EA group (*n* = 6), which were provided by Beijing Vital River Laboratory Animal Technology Co., Ltd. (Certificate number SCXK2016-0002, Beijing, China) and housed separately in the animal room (clean grade) of Institute of Acupuncture and Moxibustion, China Academy of Chinese Medical Sciences, with a temperature of 20–24°C, a humidity of (55 ± 2)%, and a circadian rhythm of 12 h/12 h. Before the experiment, rats were anesthetized with 0.65 mL/100 g i.p. of 20% urethane (Beijing Solaibao Technology Co., Ltd., China). The experimental protocol is shown in Figure 1. Rats received care consistent with the National Institutes of Health “Guide for the Care and Use of Laboratory Animals,” and the experiments were conducted in accordance with a protocol approved by the Institutional Animal Care and Use Committee of China Academy of Chinese Medical Sciences (reference no. 2015010801). All efforts were made to minimize discomfort and the number of animals used.

### 2.2. Hemodynamic Monitoring

The rat was fixed, the skin of the neck and chest was disinfected for skin preparation, the muscle and fascia were bluntly separated after the right carotid artery was exposed, an oblique small incision with a length of about 1 mm was cut, one end of PE50 catheter (Smiths Medical, UK) filled with 0.3% heparin normal saline was slowly pushed from there to the left ventricle, and the other end was connected with a pressure transducer, so that the hemodynamic change signal was input into PowerLab polygraph (AD Instruments, Australia). After the LVSP waveform was observed to be stable, the PE50 catheter was secured, and a thin layer of gauze soaked in 0.9% NaCl was covered at the surgical incision to keep it moist and clean. The baseline values of rats in each group (10 min before modeling), after modeling (after 10 min of model stabilization), and at 1, 10, 20, 40, and 60 min after intervention were monitored for LVSP, +dp/dtmax, and −dp/dtmax. The percentage is calculated as base 100%, result = each index value/base value × 100%.

### 2.3. Animal Model of Heart Failure

After the rat's basal state was stable for 10 minutes, the other groups except the NC group were first pumped into the right femoral vein of the rat with 0.4% propranolol solution (Sigma, USA) 4 mg/kg, then the flow rate was adjusted to 0.25 mg/(kg·min), and pumping continued in small doses until the end of the experiment. The animal's LVSP, +dp/dtmax, and −dp/dtmax all decreased significantly, and +dp/dtmax lower than the basic value of 60% was used as the criterion for the success of heart failure modeling. The NC group did not create a model; they only are pumped with the same dose of 0.9% NaCl as a control.

The rat model of heart failure was prepared with reference to the *Pharmacological Experiment Methodology* [8]. After the basal state of rats was stable for 10 min, except for the NC group, the other groups were pumped with 0.4% propranolol solution (Sigma, USA) into the right femoral vein of rats at a constant rate (0.2 ml/min) of 4 mg/kg by a microinjection pump (Shanghai Orcott Biotechnology Co., Ltd.), and then the flow rate was adjusted to 0.25 mg/(kg·min) for continuous low-dose pumping until the end of hemodynamic testing. The LVSP, + dp/dtmax, and −dp/dtmax of the animals were significantly decreased, and a decrease of more than 40% in +dp/dtmax was used as the criterion for successful modeling of heart failure according to the literature [9]. The NC group was not modeled, and only the same dose of 0.9% NaCl was pumped as a control.

### 2.4. Intervention Methods of Aconitine and Electroacupuncture

The dose of aconitine was set at 10 *μ*g/kg based on acute toxicological tests of the drug [10]. Aconitine (Chengdu Manster Biotechnology Co., Ltd., China) was dissolved in 0.1 mol/L HCl, adjusted to pH 7 with 1 mol/L NaOH, diluted to 300 *μ*g/mL with 0.9% NaCl solution, and filled to 50 *μ*L with 0.9% NaCl before use. After the heart failure model was stable for 10 min in the ACO group and ACO + EA group, a single bolus of aconitine solution was injected into the left femoral vein of rats using a microsyringe (Shanghai Mettler-Toledo Instrument Co., Ltd., China). While the ACO + EA group was administered, a 0.30 mm × 25 mm disposable sterile acupuncture needle (Suzhou Medical Products Factory Co., Ltd., China) was used to directly puncture the rat at “Neiguan” (PC 6, according to the textbook of experimental acupuncture, is located on forelimbs and was most frequently and effectively used to treat cardiac malfunctions including arrhythmias in clinical and experimental researches) and the left side of PC6 by 0.5 cm, with an insertion depth of about 2 mm. The ipsilateral two needle handles were connected to the positive and negative poles of the HANS-200A acupoint nerve stimulator (Nanjing Jisheng Medical Technology Co., Ltd., China), respectively. Electroacupuncture parameters are dense waves, frequency 2/15 Hz, and intensity 3 mA, for 30 min. The NC and HF groups did not receive aconitine and electroacupuncture intervention, and only 50 *μ*L 0.9% NaCl was injected as a control.

### 2.5. ECG Recording and Arrhythmia Scoring

After the onset of anesthesia, ECG electrodes were connected to the rats, and the standard limb II electrocardiogram was continuously monitored using a PowerLab multichannel physiological recorder. Observe whether there is an arrhythmia in rats at 30∼60 min after intervention, determine the type of arrhythmia, and score arrhythmia at the same time. Curtis and Walker (1988) arrhythmia scoring method [11] is shown in Table 1.

### 2.6. Echocardiographic Analysis

The structural and functional changes among the four groups were tested by Vevo2100 High Resolution Imaging Systems with a 15 MHz probe (model MS201) at 60 min after intervention (Visual Sonics, Canada). Two-dimensional cine loops and guided mode frames were recorded from the parasternal short and long axis to assess the left ventricular ejection fraction (LVEF) and the left ventricular fractional shortening (LVFS). All measured and calculated indices were presented as the average of three consecutive cardiac cycles.

### 2.7. Fluorescent Western Blotting

After the completion of the echocardiographic examination, five rats were taken from each group, the hearts were immediately harvested by thoracotomy, the excess blood was washed with 0.9% NaCl solution precooled at 4°C, and the left ventricular tissue was separated on ice, snap-frozen in liquid nitrogen, and transferred to a −80°C freezer for storage until testing. The lysis reaction solution was prepared by adding 10 *μ*L PMSF (Beijing Solaibao Co., Ltd., China) and 10 *μ*L Cocktail phosphatase inhibitor (Bimake, USA) at a ratio of 1 mL RIPA. One hundred mg of left ventricular tissue was weighed, 1 mL of lysis reaction solution was added, and the tissue was ground by a Fastprep homogenizer (MP Biomedicals, USA). After centrifugation at 4°C for 20 min at 17,949×g, the supernatant was used for protein quantification according to the instructions of BCA protein kit (Thermo, America). Proteins were transferred to 0.2 *μ*m low-background fluorescent PVDF membranes (Thermo Scientific, 22860) using an SDS electrophoresis and transfer system (Bio-Rad, America) and blocked for 1 h in 5% skimmed milk. Primary antibodies SERCA2a (1 : 500, Abcam, 2861), PLB (1 : 1000, Abcam, 2865), NCX1 (1 : 1000, Abcam, 177952), and GAPDH (1 : 1000, Cell Signaling Technology, 2118) were added after washing the membranes and incubated overnight at 4°C. After washing the membrane, fluorescent secondary antibody goat anti-mouse IgG (1 : 15000, Licor, IRDye®800CW) and goat anti-rabbit IgG (1 : 15000, Licor, IRDye®680RD) were added for 1 h at room temperature in the dark. Bands were read using an Odyssey dual-color infrared laser imaging system (Licor, USA), fluorescence values were analyzed with Image Quant TL software, and the ratio of target protein to GAPDH fluorescence values indicated the relative SERCA2a, PLB, and NCX1 protein expression content.

### 2.8. Statistical Analysis

Statistical analysis was performed using SPSS 20.0 software, and the obtained data were expressed as mean ± *SEM*. Tests for normal distribution were performed using the Shapiro–Wilk test. One-way analysis of variance (one-way ANOVA) was used to compare the means of multiple groups, and the LSD test was used for pairwise comparison. *P* < 0.05 was considered statistically significant.

## 3. Results

### 3.1. Effect of Electroacupuncture Combined with Aconitine on Hemodynamics in Rats with Heart Failure

The results are shown in Figures 2(a)–2(c). The LVSP, +dp/dtmax, and −dp/dtmax of the NC group remained relatively stable at each time point before modeling, after modeling, and 1 min, 10 min, 20 min, 40 min, and 60 min after intervention. Compared with the NC group, LVSP, + dp/dtmax, and -dp/dtmax of the HF group were decreased (*P* < 0.01), and +dp/dtmax was decreased by more than 40% at each time point after modeling and after intervention, demonstrating that the propranolol-induced heart failure model in rats was successfully prepared.

As shown in Figure 2(b), the + dp/dtmax of the ACO group and ACO + EA group increased significantly at 1 min, 10 min, 20 min, 40 min, and 60 min after the intervention (*P* < 0.01). Furthermore, the +dp/dtmax of the ACO + EA group was higher than that of the ACO group at 1 min, 20 min, 40 min, and 60 min (*P* < 0.05 or *P* < 0.01). Similar to the results shown in Figure 2(c), electroacupuncture combined with aconitine improved the -dp/dtmax of HF rats at every time point after the intervention (*P* < 0.05 or *P* < 0.01).

The above results showed that electroacupuncture combined with aconitine improved hemodynamics in rats with heart failure better than aconitine alone.

### 3.2. Effect of Electroacupuncture Combined with Aconitine on Heart Function in Rats with Heart Failure

The results are shown in Figure 3. The LVEF and LVFS of rats in the NC group were 90.26% ± 2.09% and 63.10% ± 3.33%, while the LVEF and LVFS of rats in the HF group decreased to 67.60% ± 2.04% and 39.09% ± 2.06%, respectively, which were significantly decreased compared with those in the NC group (*P* < 0.01). LVEF and LVFS of rats in the ACO and ACO + EA groups were increased to different extents compared with the HF group (*P* < 0.01), of which rats in the ACO + EA group were slightly higher than those in the ACO group, but there was no statistically significant difference. It is suggested that electroacupuncture combined with aconitine can enhance cardiac function in rats with heart failure.

### 3.3. Effect of Electroacupuncture Combined with Aconitine on the Electrocardiogram of Rats with Heart Failure

The results are shown in Figure 4. No arrhythmia occurred in the NC group during the experiment; 1 case in the HF group had atrial arrhythmia, and 1 case had occasional premature ventricular contraction with an arrhythmia score of 0.33 ± 0.21; all rats in the ACO group had different degrees of arrhythmia, of which 5 case had an occasional premature ventricular contraction and 1 case had frequent premature ventricular contraction with an arrhythmia score of 1.17 ± 0.17, which was significantly increased compared with the HF group (*P* < 0.01); while after the combination of aconitine and electroacupuncture, the incidence of arrhythmia was significantly reduced, the degree was alleviated in rats, only 1 case had an occasional premature ventricular contraction, and the arrhythmia score was 0.17 ± 0.17, which was significantly lower than that in the ACO group (*P* < 0.01), suggesting that electroacupuncture can significantly improve the side effects of aconitine in the treatment of arrhythmia in rats with heart failure.

### 3.4. Effect of Electroacupuncture Combined with Aconitine on SERCA2a and PLB Protein Expression in Rats with Heart Failure

The results are shown in Figures 5(a)–5(c). Compared with the NC group, the activity of SERCA2a in the HF group was significantly reduced, the expression of PLB was significantly increased, and the value of PLB/SERCA2a increased (*P* < 0.01). Compared with the HF group, the expression of SERCA2a protein in the ACO group did not change significantly (*P* > 0.05), the expression of PLB was weakened, and the value of PLB/SERCA2a decreased (all *P* < 0.05). Compared with the HF group and the ACO group, the ACO + EA group increased the SERCA2a protein expression, and the PLB expression decreased significantly (*P* < 0.05, *P* < 0.01). It suggests that both SERCA2a and PLB may be involved in mediating the synergistic/attenuating effect of electroacupuncture on aconitine in improving heart failure.

### 3.5. Effect of Electroacupuncture Combined with Aconitine on NCX1 Protein Expression in Rats with Heart Failure

The results are shown in Figure 5(d). The expression of NCX1 protein in the HF group was significantly higher than that in the NC group (*P* < 0.01). Compared with the HF group, there was no significant change in NCX1 protein expression in the ACO group (*P* > 0.05). The expression of NCX1 protein in the ACO + EA group was significantly downregulated compared with the HF group (*P* < 0.01), suggesting that electroacupuncture may reduce the content of NCX1 protein in myocardial tissue to achieve the synergistic/attenuated effect of aconitine in improving heart failure.

## 4. Discussion

Hemodynamic changes are the initial factor in the development of heart failure and run through the course of heart failure. Among the hemodynamic parameters monitored in this experiment, LVSP indicated that the stronger the myocardial contractility, the more sensitive the +dp/dtmax and −dp/dtmax indicators for evaluating the myocardial systolic and diastolic function, respectively; both LVEF and LVFS reflected the pumping function of the left ventricle. In this experiment, referring to the previous study [12], the heart failure model was reproduced by intravenous infusion of high-dose propranolol hydrochloride, and the hemodynamic parameters of the model rats were reduced; especially, the +dp/dtmax was reduced to less than 40%, indicating that the myocardial contractility was significantly reduced; this modeling method was simple to operate and repeatable; the success rate was more than 80%, which provided a guarantee for the relevant research on the subject.

*Fuzi* (Radix Aconiti Praeparata) is an important part of many traditional Chinese medicine prescriptions, and it has an obvious therapeutic effect on heart failure [13]. Aconitine is the main active component of Radix Aconiti Praeparata, and studies at the cellular level have shown that aconitine has a significant cardiotonic effect on heart failure models [14], but with cardiotoxicity [15]. The results of this experiment showed that the +dp/dtmax, LVEF, and LVFS of heart failure rats were significantly increased after intravenous injection of aconitine, but severe ventricular extrasystoles were induced in rats at the same time, suggesting that the efficacy and toxicity of aconitine coexist.

Acupuncture is a green therapy that is easy to operate, safe, and economical and its effect on improving heart function is definite. A large amount of relevant evidence shows that acupuncture can increase the tension of the ischemic myocardium, shorten the contraction time of myocardial fibers, increase coronary blood flow, and correct hemodynamic disorders [16]. It has also been reported that electroacupuncture at PC6 can significantly improve the heart rhythm of aconitine-induced tachyarrhythmia in rats [17]. Previous experimental results in our laboratory have shown that electroacupuncture at PC6 combined with digitalis can not only enhance the myocardial contractility of rats with heart failure but also significantly inhibit the arrhythmia caused by digitalis [18]. In view of this, we consider whether the combination of acupuncture and aconitine can improve heart failure and whether it can increase the safety of aconitine while enhancing the therapeutic effect [19]. In this study, we observed that electroacupuncture combined with aconitine significantly increased LVSP and ±dp/dtmax and also decreased arrhythmia score in rats with heart failure compared with aconitine alone. It is indicated that the immediate effect of electroacupuncture combined with aconitine improves myocardial contraction and diastolic function better, but also that electroacupuncture can significantly inhibit the toxic and side effects of arrhythmia caused by aconitine, with a certain degree of attenuation effect.

Physiologically, the concentration of [Ca^2+^]_i_ is the most critical factor for myocardial excitation-contraction coupling [20]. Recent studies have shown that abnormal calcium regulation in cardiomyocytes is the cytological basis leading to myocardial remodeling and ultimately the development of heart failure [21]; especially, SERCA2a, PLB, and NCX1 proteins play an important role in the calcium signaling pathway in cardiomyocytes. Therefore, in this study, we analyzed the specific scientific mechanism from the perspective of [Ca^2+^]_i_ regulatory proteins in cardiomyocytes on the basis of determining that electroacupuncture combined with aconitine has a synergistic and attenuated effect in improving heart failure (Table 2).

SERCA2a on SR is a key protein that regulates [Ca^2+^]_i_, which is of great significance for regulating contraction and relaxation of the heart: SERCA2a expression decreases, activity weakens, and the ability to recuperate [Ca^2+^]_i_ is impaired, making the sarcoplasmic reticulum [Ca^2+^]_i_ storage reduced, leading to a decrease in myocardial contractility and eventually developing heart failure [22]. SERCA2a has been used as an effective target for the treatment of heart failure abroad. It has been found that increasing SERCA2a gene expression in rats can improve SR calcium uptake capacity, increase SR calcium volume, and then promote calcium release so that cardiac contraction and relaxation are enhanced, while myocardial lesions due to SERCA2a gene overexpression do not occur [23]. The results of some domestic experiments showed that electroacupuncture at PC6 in rats with myocardial ischemic could significantly upregulate the expression rate of SERCA2a mRNA in cardiomyocytes, increase SERCA2a activity, inhibit calcium overload, and have a good protective effect on the myocardium [7, 24]. In this study, the content of SERCA2a in heart failure rats was significantly lower than that in normal rats, while after the intervention of aconitine, the expression of SERCA2a protein in the ACO group was not significantly different from that of the model group. However, aconitine combined with electroacupuncture could upregulate the expression of SERCA2a protein in heart failure rats. Therefore, it is considered that electroacupuncture may achieve the synergistic/attenuating effect of aconitine on improving heart failure by increasing the SERCA2a protein content in the myocardial tissue.

PLB is a small molecule sarcoplasmic reticulum membrane protein that primarily regulates the uptake and release of [Ca^2+^]_i_ by SERCA2a activity in the nonphosphorylated state [25]. Studies have shown that the dysregulation of the calcium cycle by PLB/SERCA2a is the most critical step in the process of heart failure [26]. If the expression of PLB increases and the expression of SERCA2a decreases, the ratio of PLB/SERCA2a will increase significantly, resulting in impaired SR uptake of [Ca^2+^]_i_, weakening myocardial contractility, and further promoting the occurrence and development of heart failure. There is evidence that the introduction of recombinant adenovirus carrying antisense PLB gene into adult rabbit cardiomyocytes reduces PLB protein expression, increases SERCA2a sensitivity to [Ca^2+^]_i_, significantly shortens calcium transient duration, greatly enhances myocardial contractility, and accelerates relaxation [23, 27]. The results of this study showed that the expression of PLB and the value of PLB/SERCA2a in the myocardial tissue of rats with heart failure were significantly higher than those in normal rats. The expression of PLB decreased after the intervention of aconitine, aconitine combined with electroacupuncture can further downregulate the expression of PLB, and the value of PLB/SERCA2a decreased. It indicates that PLB may be involved in mediating the protective effect of the combined application of electroacupuncture and aconitine to improve heart failure.

NCX transports 20% of [Ca^2+^]_i_ in the cytosol to the extracellular space and maintains the balance of [Ca^2+^]_i_ concentration together with SERCA2a on the SR [28]. NCX1 is an isoform of cardiac NCX protein. If NCX1 is abnormal, it will excessively excrete [Ca^2+^]_i_, affect the calcium storage in SR, cause the disorder of calcium regulation mechanism in cardiomyocytes, and ultimately trigger heart failure [29]. In this study, NCX1 protein expression in the myocardial tissue of rats with heart failure was significantly increased, indicating that NCX1 activity and expression were increased to compensate for the reduction of SERCA2a function [30, 31]. In recent years, some studies have pointed out that NCX1 inhibitors can increase SR calcium volume and thus enhance myocardial contractility by inhibiting the forward transport activity of NCX1 when used in the treatment of heart failure [32]. Aconitine has a positive inotropic effect and can induce an increase in the expression of NCX1, and a large amount of Ca^2+^ enters the cell through NCX1 to break the [Ca^2+^]_i_ balance and improve myocardial contractility while also easily inducing arrhythmias [33, 34]. Some scholars have observed that electroacupuncture can inhibit Ca^2+^ overload in cardiomyocytes and prevent the occurrence of arrhythmia [35]. In this study, the NCX1 protein expression in the ACO group was further increased compared with the HF group. However, aconitine combined with electroacupuncture could downregulate the abnormally increased NCX1 protein expression in rats with heart failure, suggesting that electroacupuncture may achieve the synergistic/attenuated effect of aconitine on improving heart failure by reducing the NCX1 protein content in myocardial tissue. However, because the role of NCX1 in the process of heart failure is diversified, the related mechanisms need to be further studied.

## 5. Conclusions

Electroacupuncture plays a synergistic and attenuated role in the effect of aconitine on improving heart failure, and the mechanism may be related to the enhancement of SERCA2a protein activity and downregulation of PLB and NCX1 protein expression in cardiomyocytes.

## Figures and Tables

**Figure 1:** The experimental protocol.

**Figure 2:** The effect of electroacupuncture combined with aconitine on LVSP (a), +dp/dtmax (b), and -dp/dtmax (c) in rats with heart failure. Data are presented as mean ± *SEM*. ^*∗∗*^*P* < 0.01 versus the NC group. #*P* < 0.05 and ##*P* < 0.01 versus the HF group. Δ*P* < 0.05 and ΔΔ*P* < 0.01 versus the ACO group (*n* = 6, each group).

**Figure 3:** M-scan of the left ventricle of rats in each group. (a) The effect of electroacupuncture combined with aconitine on LVEF and LVFS in rats with heart failure. (b) Data are presented as mean ± *SEM*. ^*∗∗*^*P* < 0.01 versus the NC group. ##*P* < 0.01 versus the HF group (n = 6, each group).

**Figure 4:** Representative traces of ECG showing the cardiac arrhythmias in the rats of different groups. (a) Arrhythmia scoring of different groups. (b) Data are presented as mean ± *SEM*. ##*P* < 0.01 versus the HF group. ΔΔ*P* < 0.01 versus the ACO group (*n* = 6, each group).

**Figure 5:** Relative expression of SERCA2a/PLB/NCX1 protein in left ventricular tissue of rats in each group. Data are presented as mean ± *SEM*. ^*∗∗*^*P* < 0.01 versus the NC group. #*P* < 0.05 and ##*P* < 0.01 versus the HF group.Δ*P* < 0.05 and ΔΔ*P* < 0.01 versus the ACO group (*n* = 5, each group).

**Table 1:** Arrhythmia scoring system.

Arrhythmia score	Type of arrhythmia
0	No arrhythmia
1	Atrial arrhythmias or occasional PVC
2	Frequent PVC
3	VT (1–2 episodes)
4	VT (>3 episodes) or VF (1–2 episodes)

**Table 2:** The variation of proteins related to calcium regulation.

Proteins	Roles played by the proteins	ACO versus HF	ACO + EA versus HF	ACO + EA versus ACO
SERCA2a	A key protein that regulates Ca^2+^ in cardiomyocytes	—	↑	↑
PLB	Inhibiting the affinity of SERCA2a to Ca^2+^	↓	↓	↓
NCX1	Exchanging Ca^2+^ inside and outside of myocardial cell membrane	—	↓	↓

↑, upregulated; ↓, downregulated; —, unchanged.

## Data Availability

The data supporting the findings of this study are available from the corresponding author upon request.

## Abbreviations

EA: Electroacupuncture
[Ca^2+^]_i_: Intracellular Ca^2+^
HF: Heart failure
NC: Normal control
ACO: Aconitine
ACO+EA: Aconitine+electroacupuncture
VF: Ventricular fibrillation
VT: Ventricular tachycardia
PVC: Premature
LVSP: Left ventricular systolic pressure
±dp/dtmax: Maximal rate for left ventricular pressure rising and declining
LVEF: Left ventricular ejection fraction
LVFS: Left ventricular fractional shortening
SERCA2a: Sarcoplasmic/endoplasmic reticulum Ca^2+^ ATPase
PLB: Phospholamban
NCX: Na^+^-Ca^2+^ exchange
SR: Sarcoplasmic reticulum
